# Genetic variations in E6, E7 and the long control region of human papillomavirus type 16 among patients with cervical lesions in Xinjiang, China

**DOI:** 10.1186/s12935-019-0774-5

**Published:** 2019-03-20

**Authors:** Xiangyi Zhe, Huizhen Xin, Zhenzhen Pan, Fuyuan Jin, Weinan Zheng, Hongtao Li, Dongmei Li, Dongdong Cao, Ying Li, Chunhe Zhang, Shaowei Fu, Renfu Shao, Zemin Pan

**Affiliations:** 1 Key Laboratory of Xinjiang Endemic and Ethnic Diseases/Department of Biochemistry and Molecular Biology, School of Medicine, Shihezi University, Shihezi, 832002 Xinjiang China; 2 Xinjiang Production and Construction Corps of the Fourth Division Hospital, Yining, 835000 Xinjiang China; 3 School of Science and Engineering, Genecology Research Centre, The Animal Research Centre, University of the Sunshine Coast, Sippy Downs, QLD 4556 Australia

**Keywords:** Human papillomavirus, Cervical cancer, Genetic variations, Polymorphism analysis, Phylogenetic tree

## Abstract

**Background:**

Xinjiang is one of the areas with the highest incidence of cervical cancer in China. Genetic variation in Human papillomavirus type 16 (HPV16) may increase the ability of the virus to mediate carcinogenesis and immune escape, which are risk factors for the progression of cervical cancer. We investigated polymorphism in HPV16 and the distribution of its sub-lineages in the region by analyzing the *E6*, *E7* and *long control region* (*LCR*) gene sequences from women with HPV16-positive cervical samples in Xinjiang.

**Methods:**

A total of 138 cases of cervical lesions and squamous cell carcinoma with infection of HPV16 virus were collected. The *E6* and *E7* genes and *LCR* of HPV16 virus were sequenced and compared with the HPV16 European prototype reference and other HPV16 mutants for single nucleotide polymorphisms. Neighbor-joining phylogenetic trees were constructed using E6, E7 and LCR sequences.

**Results:**

Fourteen missense mutations were found in the *E6* gene; the loci with the highest mutation frequency were T350G (36/75, 48%) and T178G (19/75, 25.3%). In the *E7* gene, the locus with the highest mutation frequency was A647G (18/75, 24%). A total of 33 polymorphic sites were found in the *LCR*, of which T7447C (39/95, 40.1%) was the most frequent.

**Conclusion:**

HPV16 in Xinjiang is mainly of the European variant, followed by the Asian variant type; no Africa 1, 2 or Asia–America variant types were found.

## Background

Cervical cancer is the second most common malignant disease after breast cancer among women globally and has been ranked fourth among cancer-related deaths. The newly diagnosed cases in China (130,000) account for about a quarter of those in the world (approximately half a million). Cervical cancer is the most common malignant tumor of the female reproductive tract and has a major impact on women’s health and life expectancy [1]. Epidemiological data have confirmed that persistent infection with high-risk human papillomavirus (HR-HPV) (such as HPV16 and HPV18) can lead to atypical hyperplasia and cancer in the cervix, thus confirming HPV as a central cause of this malignant tumor [2]. Xinjiang is one of the areas with the highest incidence of cervical cancer in China, most of which is closely related to HPV16 infection [3]. The production of cervical cancer by HPV is mainly mediated by the *E6* and *E7* genes [4]. In addition, the E1 protein promotes viral genome replication and the E2 protein is negatively correlated with oncogene expression. The integration and mutation of E1 and E2 may promote the expression of virus genes *E6* and *E7*, thus leading to the occurrence and development of cervical cancer [5]. E7 is an oncoprotein with high carcinogenic risk containing 98 amino acids, which makes epithelial cells immortal with the cooperation of HPV E6 protein [6].

Many researchers have sequenced the HPV16 genes isolated from cervical lesions. It has been found that the variation in HPV16 *E6* and *E7* is correlated with the progression of cervical lesions and that HPV16 variant and HPV16 *E6* and *E7* mutations vary by racial and geographic area [7–9].

A meta-analysis was reported in 2013 by Comet et al. [10], using the scope of cancer caused by HPV16 all over the world, which showed that the European (Eur) variant is the most common sub-lineage and may be associated with persistent infection by HPV and increased risk of the progression of cervical lesions. By contrast, the results of Sun et al. [11] in the Liaoning province of China show that the Eur variants are negatively correlated with the severity of cervical disease at a level of cervical intraepithelial neoplasia 2/3 (CIN 2/3) or higher. In that study, Asian (As) variants were found in precancerous lesions and cases of cervical cancer, and were associated with disease progression. In addition, epidemiological studies have suggested that Asia–America (AA) variants can promote continuous infection with HPV and disease progression [12]. Smith [13] and Berumen [14], in Costa Rica and Mexico, have reported that both AA and North America (NA) variants can increase the risk of CIN 3 cervical cancer in women. At the same time, they opined that variation can increase the ability of keratinocytes to achieve in vitro transformation. Overall, different HPV variants are associated with severity of cervical lesion. The variations of the HPV16 gene sequence may increase the virulence of the virus and mediate immune escape, which are risk factors for cervical cancer progression. However, different studies have inconsistent results, which may be related to differences in the genetic background of local populations.

Our study was designed to analyze the *E6*, *E7*, and *long control region* (*LCR*) gene sequences of HPV16-positive cases of cervical disease in the female population of Xinjiang, to investigate polymorphism of the HPV16 sub-lineages and their distribution in the local area. We explored the relationships between HPV16 *E6*, *E7*, and *LCR* gene mutations and the incidence of cervical cancer in Xinjiang, to accumulate molecular epidemiological data for the study of HPV16 gene polymorphism in cervical lesions.

## Materials and methods

### Specimen collection

Primers for HPV16 E6 were used to screen samples from women with cervical lesions or those who had undergone surgery for cervical squamous cell carcinoma, and biopsy samples. The participants attended the Friendship Hospital (in 2016), or the People’s Hospital of Kashi (southern Xinjiang, China) and the People’s Hospital of Autonomous region (northern Xinjiang, China) during 2011–2014. Cases were confirmed by pathological examination and identified as cervical squamous cell carcinoma. A total of 138 cases of cervical lesions and squamous cell carcinoma with HPV16 infection were obtained. None of the patients had a history of long-term residence in other places. The samples were stored at − 80 °C for further processing. Informed consent was obtained from all patients and the study protocol was reviewed and approved by the ethics committees of the hospitals.

### DNA extraction and HPV16 identification

DNA extraction was carried out using an SK1252 genomic DNA extraction kit (Shanghai Sangon Biological Engineering Technology and Services Company, Shangai, China) according to the instructions of the kit. The HPV16 E6 primers were designed and polymerase chain reaction (PCR) was used to detect HPV16 virus. The primer sequences for identification of HPV16 E6 were: HPV16 E6-F: 5′-gacccagaaagttaccacag-3′, HPV16 E6-R: 5′-cacaacggtttgttgtattg-3′ (F, forward primer; R, reverse primer).

### PCR amplification and sequencing

The HPV16 E6, E7 and LCR gene fragments were amplified by PCR. Each 50-µL PCR reaction mixture contained 20 pmol of each primer, 50 mM KCl, 2.5 mM MgCl_2_, 100 mM Tris–HCl, pH 8.3, 0.1% Triton X-100, 50 µM of each dNTP, 1.8 U of HotStar Taq polymerase (QIAGEN, Hilden, Germany) and 5 µL template DNA. The PCR reaction conditions were as follows: 94 °C for 5 min; 30 cycles of 55 °C for 45 s, 72 °C for 60 s, 94 °C for 15 s; 55 °C for 45 s, 72 °C for 5 min. The sequencing primers are shown in Table 1.

**Table 1:** Information on primers

	Primer name	Primer sequence	Gene area covered (bp)
E6/E7	16E6-15N	5′-AAACTAAGGGCGTAACCGAAATC-3′	44–910
	16E7-16C	5′-CAGCCTCTACATAAAACCATCCAT-3′	
	16E6-13N	5′-AACCGAAATCGGTTGAACCG-3′	60–857
	16E7-13C	5′-TGCAGGATCAGCCATGGTAGAT-3′	
LCR/E6	LCR-F	5′-ACGCAAAAAACGTAAGCTG-3′	7152–546
	E6-R-2	5′-TCCATGCATGATTACAGCTGGGTT-3′	
	LCR-F	5′-ACGCAAAAAACGTAAGCTG-3′	7152–230
	16LCR-E6-5C	5′-ATCCCGAAAAGCAAAGTCAT-3′	

*N* normal strand, *C* complementary strand

### Phylogenetic analysis of HPV16 variants

The PCR products were purified using SAP (Promega) and Exo I (Epicentre) and sequenced directly using an ABI Big-Dye Terminator v3.1 Cycle Sequencing Kit on a DNA analyzer (ABI3130XL) at Genesky Biotechnologies Inc (Shanghai, China). Single nucleotide polymorphisms (SNP) were analyzed using Polyphred and were aligned with the European prototype (GenBank: NC_001526.2) [15] and other typical HPV16 variants including As (GenBank: AF534061; AB889492), Af-1 (GenBank: AF472508; HQ644238), AA (GenBank: AF402678) and AA1 (GenBank: HQ644247) for comparison. A phylogenetic tree was built using MEGA 6 [16] (Fig. 1).

**Fig. 1:** Phylogenetic tree analysis of the HPV16 E6/E7 gene. Phylogenetic tree constructed from E6 and E7 nucleotide sequences of 75 HPV16 variants. The red branches (n = 18) belong to Asian strains; the remainder of the branches (n = 57) belong to European strains. Study sequences are labeled in XJ numbers, others are reference GenBank sequences. Phylogenetic trees were constructed by the neighbor-joining (NJ) method and the Kimura 2-Parameter model with bootstrap resampling (1000 replicates) by the MEGA 6 package. Values lower than 50% are not shown

## Results

### Mutation analysis of HPV16 E6, E7 and LCR genes

In total, 138 HPV16 positive samples were sequenced to give full-length HPV16 LCR sequences, and 90 cases were chosen to carry out full-length HPV16 *E6* and *E7* gene sequencing. Finally, 75 E6 and E7 sequences and 95 LCR sequences were obtained. The HPV16 prototype (European prototype, GenBank accession: NC_001526.2) was used as the standard for comparison, and the gene polymorphism sites are shown in Tables 2 and 3.

**Table 2:** Nucleotide sequence variations in E6 and E7 of HPV16 (n = 75)

		E6 base sites									
HPV16 variants:		T109C	A131C	C168G	G176A	*T178G*	T178A	T183G	A275G	A276G	T295G
AA changes:				T22S	D25N	*D25E*	D25Q	I27R	N58D	N58S	D64E
E reference:		T	A	C	G	T	T	T	A	A	T
AA:		T	A	C	G	T	T	T	A	A	T
As:		T	A	C	G	G	G	T	A	A	T
Af:		T	A	C	G	T	T	T	A	A	T
Mutation:		1/75	1/75	1/75	1/75	19/75	1/75	2/75	1/75	1/75	1/75
Ep	11										
Ep	3										
Ep	2							G			
Ep	2										
Ep	1						A			G	
Ep	1										
Ep	1				A						
E-350G	30										
E-350G	1										
E-350G	1	c									
E-350G	1										
E-350G	1										G
E-350G	1								G		
E-350G	1			G		G					
As	15					G					
As	2					G					
As	1		c			G					

		E6 base sites					E7 base sites				
HPV16 variants:		*T350G*	C360A	A442C	A645C	A646C	*A647G*	*G666A*	*T760C*	*T846C*	
AA changes:		*L83V*	T86K	E113	L28F	N29H	*N29S*				
E reference:		T	C	A	A	A	A	G	T	T	
AA:		G	C	A	A	A	A	G	T	T	
As:		T	C	A	A	A	G	G	T	C	
Af:		T	C	A	A	A	A	G	T	T	
Mutation:		36/75	1/75	1/75	1/75	1/75	18/75	4/75	4/75	3/75	
Ep	11										
Ep	3								c		
Ep	2										
Ep	2							a			
Ep	1							a			
Ep	1							a			
Ep	1								c		
E-350G	30	G									
E-350G	1	G		C	C						
E-350G	1	G									
E-350G	1	G									
E-350G	1	G	A								
E-350G	1	G									
E-350G	1	G				C					
As	15						G				
As	2						G			c	
As	1						G			c	

Bolditalic are the most common mutation sites

Capital letters indicate variants with an amino acid change, lower-case letters indicate silent mutations

*AA change* amino acid change, *Ep* European prototype, *AA* Asian–American lineage, *As* Asian lineage, *Af* African lineage

**Table 3:** Nucleotide sequence variations in the LCR of HPV16 (n = 95)

	n = 95	LCR base sites														
HPV16:		*T*	A	A	*C*	*A*	A	C	A	C	T	A	T	*T*	G	*T*
		*7*	7	7	*7*	*7*	7	7	7	7	7	7	7	*7*	7	*7*
		*1*	2	2	*2*	*2*	2	3	3	3	4	4	4	*4*	6	*7*
Variants:		*9*	3	5	*6*	*8*	8	0	2	9	0	1	3	*4*	9	*1*
		*9*	1	3	*8*	*5*	7	8	3	3	4	7	8	*7*	9	*1*
		*C*	C	G	*T*	*C*	C	T	C	T	G	G	G	*C*	A	*G*
E reference:		T	A	A	C	A	A	C	A	C	T	A	T	T	G	T
AA:		T	C	A	C	A	A	C	A	T	T	A	T	T	G	T
As:		C	C	A	T	C	C	C	A	C	T	A	T	T	G	T
Af:		T	A	A	C	A	A	C	A	C	T	A	T	T	G	T
Mutation:		*16*	2	1	*16*	*16*	11	1	1	1	1	9	1	*39*	3	*16*
Ep-350T	16															
Ep-350T	2															
Ep	2															
Ep	1															
Ep	1	C														
Ep	1	C						T		T						
Ep	1															
E-T7711G	15															G
E-T7711G	1										G					G
E-T7447C	27													C		
E-T7447C	7													C		
E-T7447C	3													C	A	
E-T7447C	1													C		
E-T7447C	1													C		
As	9	C			T	C	C					G				
As	2	C			T	C										
As	2	C			T	C										
As	1	C			T	C	C		C							
As	1	C		G	T	C	C									
As	1	C			T	C							G			

	n = 95	LCR base sites														
HPV16:		*A*	T	G	G	T	G	C	*G*	G	A					
		*7*	7	7	7	7	7	7	*7*	7	7	C	*C*	A	C	
		*7*	7	7	8	8	8	8	*8*	8	8	1	*2*	4	7	
Variants:		*2*	7	9	0	2	3	3	*3*	6	7	3	*4*	1	3	
		*7*	8	6	3	4	1	7	*9*	6	1	T	*T*	C	T	
		*C*	C	A	A	C	C	T	*A*	A	G					
E reference:		A	T	G	G	T	G	C	G	G	A	C	C	A	C	
AA:		A	T	G	G	T	G	C	G	G	A	C	C	A	C	
As:		C	C	G	G	T	G	C	A	G	A	C	T	A	C	
Af:		A	T	G	G	T	T	C	G	A	A	C	C	A	C	
Mutation:		*16*	1	3	1	3	1	1	16	7	2	3	*16*	2	2	
Ep-350T	16															
Ep-350T	2														T	
Ep	2					C						T		C		
Ep	1						C									
Ep	1															
Ep	1															
Ep	1					C										
E-T7711G	15															
E-T7711G	1															
E-T7447C	27															
E-T7447C	7									A						
E-T7447C	3			A												
E-T7447C	1				A											
E-T7447C	1											T				
As	9	C							A				T			
As	2	C							A		G		T			
As	2	C							A				T			
As	1	C						T	A				T			
As	1	C	C						A				T			
As	1	C							A				T			

Bolditalic are the most common mutation sites

*Ep* European prototype, *AA* Asian American lineage, *As* Asia lineage, *Af* African lineage

Nineteen single nucleotide changes were identified among the sequencing results for E6 and E7, including 14 missense mutations and five synonymous mutations: 11/14 missense mutations were distributed in the E6 gene (C168G, G176A, T178G, T178A, T183G, A275G, A276G, T295G, T350G, C360A and A442C) and 3/14 missense mutations (A645C, A646C, A647G) were located in the E7 gene. These caused the amino acid to change from threonine to serine (T22S), aspartic acid to asparagine (D25N), aspartic acid to glutamic acid (D25E), aspartic acid to glutamine (D25Q), isoleucine to arginine (I27R), asparagine to aspartic acid (N58D), asparagine to serine (N58S), aspartic acid to glutamic acid (D64E), leucine to valine (L83V), threonine to lysine (T86K), glutamic acid to aspartic acid (E113D), leucine to phenylalanine (L28F), asparagine to histidine (N29H) and asparagine to serine (N29S), respectively. The two synonymous mutations of the E6 gene were nt109 (T to C) and nt 131 (A to C). The most common mutation sites in HPV16 E6 were T350G (36/75, 48%) and T178G (19/75, 25.3%). Compared with E6, the E7 gene is more conserved; the most common mutation site in E7 was A647G (18/75, 24%), and only one sample of A645C and A646C showed mutation. Notably, 18 cases of the A647G mutation were combined with the T178G mutation, and we considered that the A647G of E7 and T178G of E6 were co-variations.

Among the results of LCR sequencing, 33 polymorphic sites were found (the Table lists only 29 sites), of which four polymorphic sites (G7191T, nt7432–7433:GC to CGG, G7518A and A7861 deletions) showed 100% mutation in 95 samples. The remaining 29 mutations were mainly T7447C (39/95, 40.1%), followed by T7199C (16/95, 16.8%), C7268T (16/95, 16.8%), A7285C (16/95, 16.8%), T7711G (16/95, 16.8%), A7727C (16/95, 16.8%), G7839A (16/95, 16.8%) and C24T (16/95, 16.8%). We also found that six loci, T7199C, C7268T, A7285C, A7727C, G7839A, and C24T, in the LCR sequence were possibly co-variations.

### Phylogenetic tree analysis

Phylogenetic analysis used the neighbor-joining method and the Kimura 2-Parameter model with bootstrap resampling (1000 replicates) of Mega 6 to construct the phylogenetic tree. Bootstrap values > 95% indicate very high confidence; 75–94%: high confidence; 50–74%: low confidence; and < 50%: no confidence. The bootstrap values (≥ 50%) are indicated in internal nodes.

The results of the phylogenetic analysis of E6 and E7 (Fig. 1) showed that, among the 75 samples, 18 samples (bootstrap values = 77%) belonged to As and the remaining 57 samples (bootstrap values = 99%) belonged to Eur strains.

The LCR phylogenetic analysis result (Fig. 2) showed that, among the 95 samples, only 16 of the samples (bootstrap values = 86%) belonged to As; Af-1, Af-2 and AA strains were not found.

**Fig. 2:** Phylogenetic tree analysis of the HPV16 LCR gene. Phylogenetic tree constructed from LCR nucleotide sequences of 95 HPV 16 variants. The red branches (n = 16) belong to Asian strains, the rest of the branches (n = 79) belong to European strains. Study sequences are labeled in XJ numbers; others are reference GenBank sequences. Phylogenetic trees were constructed by the neighbor-joining (NJ) method and the Kimura 2-Parameter model with bootstrap resampling (1000 replicates) by the MEGA 6 package. Values lower than 50% are not shown

### Distribution of HPV16 sub-lineages in different histopathological grades

According to the E6 and E7 sequences, the HPV16 in our study could be divided into the Ep, E-350G and As sub-lineages. Use of the Pearson Chi squared test or Fisher’s exact test on the distribution of the three sub-lineages in different histological grades (considering P < 0.05 as statistically significant), showed that in different histological grades, the distributions of the three sub-lineages were significantly different when comparing normal with CIN 1 and CIN 2/3 (*P *= 0.001), or CIN 2/3 with cervical cancer (*P *= 0.023) (Table 4). The analysis showed no significant difference in the distribution of the sub-lineages of the HPV16 LCR sequence (*P* > 0.05) (Table 5).

**Table 4:** Distribution of sub-lineages of HPV16 E6, E7 (n = 75) according to the histopathological results

Histology		Ep		E-350G		As	
		n	%	n	%	n	%
Normal or CIN1	15	6	40.0	3	20.0	6	40.0
CIN2/3	19	1	5.3	15	78.9	3	15.8
Cervical cancer	41	13	31.7	17	41.5	11	26.8
*P-*value				*0.007*			

Italic value indicates statistically significant

*CIN* cervical intraepithelial neoplasia, *P* Pearson chi-square test or Fisher’s exact test

Comparison between normal and CIN 1 or CIN 2/3, *P* = 0.001

Comparison between CIN 2/3 and cervical cancer, *P* = 0.023

Comparison between Normal or CIN 1 and cervical cancer: *χ*^2 ^= 2.267, *P *= 0.322

**Table 5:** Distribution of sub-lineages of HPV16 LCR (n = 95) according to the histopathological results

Histology		Ep		E-T7447C		E-T7711G		As	
		n	%	n	%	n	%	n	%
Normal or CIN1	17	5	29.4	6	35.3	3	17.6	3	17.6
CIN2/3	18	5	27.8	7	38.9	2	11.1	4	22.2
Cervical cancer	60	14	23.3	26	43.3	11	18.3	9	15.0
*P-*value					0.961				

*CIN* cervical intraepithelial neoplasia

*P*-value was calculated using Fisher’s exact test

## Discussion

A large number of experiments have been conducted to study the mutation of a variety of high-risk human papillomaviruses, concentrating mainly on HPV16, 18, 33, 35, and 45. However, HPV16 is the primary pathogenic factor in the occurrence of cervical cancer, and therefore most reports are related to HPV16 variation. They indicate that mutation of the virus may lead to the substitution of amino acids in the corresponding encoded proteins, which can alter the biological characteristics and immunogenicity of the virus, and affect the carcinogenic ability of HPV16 [17]. HPV16 gene variation shows a degree of regionality and it is divided it into six main branches according to geographic location: Eur, As, AA, Af-1, Af-2 and NA [10, 18]. In addition, Eur viruses have been divided into a few small branches, such as E-T350 (Ep), E-G350 (T350G), E-G131 (A131G) and E-C109 (T109C). Each study of genetic variation in HPV16 has shown that a particular gene locus mutation will allow the virus to escape more easily from the monitoring of the host immune system or increase the opportunity of secondary virus infection, or cause cells to be malignant.

In this study, a total of 13 polymorphic sites were identified in 75 HPV16 E6 sequences, and T350G (36/75, 48%) and T178G (19/75, 25.3%) comprised the majority of 11 missense mutations, this result is consistent with that of Cai et al. [19]. Studies have shown that HPV16 *E6* T350G (L83V) variants are prevalent in high cervical lesions in Moroccan women and are closely related to the progression of cervical cancer [20]. T178G (D25E) variations are mainly distributed in the Asian population (such as China, Japan and South Korea) [21, 22]; the mutation can interact with *Human Lymphocyte Antigen (HLA)* gene polymorphisms and promote the development of cervical cancer. Chansaenroj et al. [23] also suggest this mutation can increase the likelihood of persistent viral infection and cervical cancer progression.

The results of this study show that the common polymorphism site of the *E7* gene is A647G, which is similar to the results of Yang et al. [24]. Interactions between the *E7* gene and tumor suppressor protein Rb are widely considered to be one of the main causes of cervical cancer. Amino acids 21–34 of the E7 protein form a region that combines with tumor suppressor protein Rb [25], and the A647G mutation may block the physiological function of Rb, thereby maintaining long-term infection with HPV. In addition, most of the mutations in A647G occur in the As sub-lineage. Further studies are needed to determine whether the mutation leads to the higher carcinogenicity of the As sub-lineage. It was found that A645C (L28F) has an incidence of 19% in cervical cancer tissues from Korean women [26] and that this mutation also occurs in Italy and Japan [27, 28]. However, only one mutation was found in our study, further emphasizing that HPV mutation has regional characteristics.

Most studies aim only to investigate whether there is a combination of mutations within individual genes, and there are relatively few reports of multiple genes with joint mutations. However, it has been reported that joint mutation of *E6* T350G and *E7* A647G may be Chinese specific [21]. In contrast to the above report, 36 cases of T350G polymorphism were found in this study, and there was no polymorphism of the joint site mentioned above. Among 19 samples with polymorphism in *E6* T178G or *E7* A647G, 18 cases (94.7%) had two loci changed at the same time, which was consistent with the studies of Ding [29]. In addition, three cases showed the *E7* T846C mutation in association with the combined mutation of the above two loci. The effect of these joint mutations on the carcinogenicity of HPV remains to be further studied.

The LCR is the most variable region of the HPV16 genome, and may exert a vital function in persistent virus infection and the progression of cervical cancer. It contains the sequences associated with transcriptional regulation, and it is also the replication origin of HPV [8, 30]. Accounting for 100% of all infections, G7191T and G7518A mutations, were predicted by Xi et al. [31] to be, respectively, the binding sites for FOXA1 (Forkhead box protein A1), which is involved in the regulation of breast cancer, liver cancer, prostate cancer, lung cancer and endometrial cancer, and for SOX9 (sex-determining region Y-box 9), which is the potential cervical cancer tumor suppressor that, through the activation of p21^WAF1/CIP1^, inhibits cervical cancer cell growth. The frequency of A7727C mutation is relatively high. It may be the binding site of transcription factor PHOX2A (paired-like homeobox 2a), which is involved in cell proliferation and lung cancer metastasis.

The phylogenetic tree of the E6 and E7 sequences constructed using MEGA 6 shows that the prevalent strains of HPV16 in the Xinjiang area were mainly of the Eur (57/75, 76%), followed by the As (18/75, 24%); no Af-1 or Af-2 and AA variant types were found. The same conclusion was obtained in the analysis of the LCR sequences. Some of these branches had lower bootstrap values and may be associated with mutations in certain sites. As discussed above, the Eur variant of HPV16 is the most common sub-lineage in Xinjiang. In this study, we found that the association of HPV16 sub-lineages with different histopathological grades was statistically significant (*P *= 0.007). Future studies will be conducted to explore the role of HPV16 variants in the development of cervical cancer, based on a larger sample size, and will involve in vitro cell culture.

The HPV vaccine has become a research hotspot, including therapeutic vaccination for individuals infected with HPV virus and those with genital tract disease caused by HPV. Compared with prophylactic vaccines, therapeutic vaccines are mainly targeted against antigenic determinants of HPV early proteins, E6 or E7. E6 and E7 are the main transforming genes: cervical cancer cells cannot evade the immune response because of the absence of antigens, so E6 and E7 proteins can be used as targets for therapeutic vaccines against cervical cancer. However, HPV virus vaccine is highly specific; there are differences in immunogenicity among different HPV16 types, thus increasing the difficulty in the development of therapeutic vaccines. Therefore, the investigation and analysis of different HPV16 variants in the population of specific regions has significance in uncovering the carcinogenic mechanism of HPV16 and in developing preventive and therapeutic vaccines against HPV.

## Conclusion

Samples of HPV16 in Xinjiang were mainly of the European variant, followed by the Asian variant; no African 1, 2 or Asia–America variant types were found.
